RETRACTED

# Neuropilin-1^high^CD4^+^CD25^+^ Regulatory T Cells Exhibit Primary Negative Immunoregulation in Sepsis

**DOI:** 10.1155/2016/7132158

**Published:** 2016-04-27

**Authors:** Yu-Lei Gao, Yan-Fen Chai, An-Long Qi, Ying Yao, Yan-Cun Liu, Ning Dong, Li-Jun Wang, Yong-Ming Yao

**Affiliations:** ^1^Department of Emergency Medicine, Tianjin Medical University General Hospital, Tianjin 300052, China; ^2^Trauma Research Center, First Hospital Affiliated to the Chinese PLA General Hospital, Beijing 100048, China; ^3^State Key Laboratory of Kidney Disease, The Chinese PLA General Hospital, Beijing 100853, China

## Abstract

Regulatory T cells (Tregs) appear to be involved in sepsis-induced immune dysfunction; neuropilin-1 (Nrp-1) was identified as a surface marker for CD4^+^CD25^+^Tregs. In the current study, we investigated the negative immunoregulation of Nrp-1^high^CD4^+^CD25^+^Tregs and the potential therapeutic value of Nrp-1 in sepsis. Splenic CD4^+^CD25^+^Tregs from cecal ligation and puncture (CLP) mouse models were further segregated into Nrp-1^high^Tregs and Nrp-1^low^Tregs; they were cocultured with CD4^+^CD25^−^  T cells. The expression of forkhead/winged helix transcription factor-3 (Foxp-3), cytotoxic T-lymphocyte associated antigen-4 (CTLA-4), membrane associated transforming growth factor-*β* (TGF-β^m+^), apoptotic rate, and secretive ability [including TGF-*β* and interleukin-10 (IL-10)] for various types of Tregs, as well as the immunosuppressive ability of Tregs on CD4^+^CD25^−^  T cells, were determined. Meanwhile, the impact of recombinant Nrp-1 polyclonal antibody on the demethylation of Foxp-3-TSDR (Treg-specific demethylated region) was measured in* in vitro* study. Sepsis* per se* markedly promoted the expression of Nrp-1 of CD4^+^CD25^+^Tregs. Foxp-3/CTLA-4/TGF-β^m+^ of Nrp-1^high^Tregs were upregulated by septic challenge. Nrp-1^high^Tregs showed strong resilience to apoptosis and secretive ability and the strongest immunosuppressive ability on CD4^+^CD25^−^  T cells. In the presence of lipopolysaccharide (LPS), the recombinant Nrp-1 polyclonal antibody reduced the demethylation of Foxp-3-TSDR. Nrp-1^high^Tregs might reveal primary negative immunoregulation in sepsis; Nrp-1 could represent a new potential therapeutic target for the study of immune regulation in sepsis.

## 1. Introduction

Sepsis is still a leading cause of death among critical patients in the intensive care units, and the life quality of the survivors would usually be impaired [1–5]. There was a serious decrease of immunocytes, including B/T-lymphocytes, dendritic cells (DCs), gastrointestinal epithelial cells, and even thymocytes, at the beginning of sepsis as shown in both animal models and septic patients [6–9]. It has been noted that the septic patients would gradually enter immunosuppression after primary hyperinflammatory response, which is defined as immunoparalysis [2, 4, 6, 7]. In recent years, investigators have become interested in the study of the mechanisms regarding immunosuppression and the development of new methods to regulate immune response during sepsis, including both activation of Tregs and apoptotic depletion of immunocytes [10].

RETRACTED

As a class of CD4^+^ T cell subsets, Tregs are a group of specialized immune cells that play an important role in immune homeostasis [11]. During the development of sepsis, Tregs subdue inflammation and tissue damage, and they may also cause immune dysfunction, such as induction of T-lymphocytic apoptosis, inhibition of CD4^+^/CD8^+^ T-lymphocytic function, and mediation of shifting from the helper T cell 1 (Th1) to Th2 response, especially immunoparalysis via expression of CTLA-4 and TGF-*β* ^m+^, as well as anti-inflammatory cytokines (IL-10 and TGF-*β*) [12–17].

Nrp-1 is characterized as a single-pass transmembrane glycoprotein, which is originally described to be involved in axon guidance, revascularization, and tumorous growth [18, 19]. Recently, Nrp-1, an essential component of the immunological response in humans and animals, is identified as a potent surface marker for CD4^+^CD25^+^Tregs [20–23]. In addition, the expression of Nrp-1 on Tregs was correlated with the expression of Foxp-3 and suppressive capacity [24]. Solomon and his colleagues further showed that Nrp-1^+^CD4^+^CD25^+^Tregs suppressed the proliferation of CD4^+^CD25^−^ T cell more efficiently than CD4^+^CD25^+^Tregs and Nrp-1^−^CD4^+^CD25^+^Tregs in a mouse model of experimental autoimmune encephalomyelitis (EAE) [25]. In our previous study, we indicated that tuftsin-derived T-peptide, the typical ligand of Nrp-1, had the ability to improve the outcome of septic mice in a dose- and time-dependent manner and was associated with downregulation of the negative immunoregulation of Tregs and improvement of the microenvironment of cellular immunosuppression in septic mice [26]. Thus, further investigation on the impact of Nrp-1 on the negative immunoregulation of Tregs will provide a new target for the study of immune regulation in sepsis.

In the present study, the objective, using the classical septic model, that is, CLP, is to investigate the impact of sepsis on the expression of Nrp-1 on CD4^+^CD25^+^Tregs and the negative immunoregulation of Nrp-1^high^CD4^+^CD25^+^Tregs in septic mice, as well as the potential therapeutic value of Nrp-1 in sepsis. We demonstrated that the expression of Nrp-1 on CD4^+^CD25^+^Tregs was significantly upregulated in a grade- and time-dependent manner, Nrp-1^high^CD4^+^CD25^+^Tregs possessed primary negative immunoregulation in septic response, and recombinant Nrp-1 polyclonal antibody markedly downregulated the demethylation of Foxp-3-TSDR in the stimulation of LPS in a dose-dependent manner. Nrp-1 could represent a new potential therapeutic target for the study of immune regulation in sepsis.

RETRACTED

## 2. Materials and Methods

### 2.1. Animals

Inbred male BALB/c mice (Laboratory Animal Center of Chinese Academy of Medical Sciences, number SCXK-Jing-2009-0007, Beijing, China), aged 6–8 weeks, weighing 20 ± 2 g, were used in the present study. All procedures were undertaken in accordance with the criteria of National Institute of Health Guide for the Care and Use of Laboratory Animal and approved by the Scientific Investigation Board, Medical College of Chinese PLA, Beijing, China.

### 2.2. Medium and Reagents

The medium used throughout the* in vitro* experiment was RPMI1640 (containing 100 U/mL penicillin, 100 *μ*L/mL streptomycin, and 1.5 mM glutamine) with 10% heat-inactivated fetal bovine serum (FBS). CD4^+^CD25^+^ regulatory T cell isolation kits, goat anti-rabbit IgG microbeads, rabbit anti-mouse Nrp-1, and LD/SM columns were purchased from Miltenyi Biotec GmbH, Bergisch Gladbach, Germany. Cell counting kit-8 (CCK-8) was purchased from Dojindo, Kumamoto, Japan. Fluorescein isothiocyanate- (FITC-) conjugated annexin-V apoptotic kit was purchased from Nanjing Keygen Biotech, Nanjing, China. Purified hamster anti-mouse CD3e and CD28 were purchased from BD Pharmingen, San Diego, CA. Antibodies used for flow cytometric analysis, including FITC-conjugated anti-mouse/rat-Foxp-3, FITC-conjugated anti-mouse CD152 (CTLA-4), and allophycocyanin- (APC-) conjugated anti-mouse/rat-TGF-*β* ^m+^, were purchased from eBioscience, San Diego, CA. APC-conjugated anti-mouse/rat-Nrp-1 and recombinant Nrp-1 polyclonal antibody were purchased from R&D Systems, Minneapolis, MN. Enzyme-linked immunosorbent assay (ELISA) kits for interferon-*γ* (IFN-*γ*), IL-2, IL-4, IL-10, and TGF-*β* were purchased from Excell Biol, Shanghai, China. Ketamine and Su-Mianxin-II (containing 2,4-xylazole, ethylenediaminetetraacetic acid, dihydroetopine, and haloperidol) were purchased from China Academy of Military Medical Sciences, Beijing, China, and they were used as the anesthesia for animals.

### 2.3. Isolation of Splenic CD4^+^CD25^+^Tregs, CD4^+^CD25^−^ T Cells, Nrp-1^high^CD4^+^CD25^+^Tregs, and Nrp-1^low^CD4^+^CD25^+^Tregs

Spleens were harvested and prepared into single cell suspension by passing through a 30 *μ*m stainless steel mesh twice and then treated with Ficoll-Paque density gradient centrifugation. CD4^+^CD25^+^Tregs and CD4^+^CD25^−^ T cells were isolated from mononuclear cells using mouse CD4^+^CD25^+^Treg isolation kit and MiniMACS*™* separator (Miltenyi Biotec GmbH, Bergisch Gladbach, Germany) according to manufacturer's instructions. CD4^+^CD25^+^Tregs were incubated with a rabbit anti-mouse Nrp-1 antibody (Abcam, Cambridge, MA) for 20 minutes at 4°C, washed and incubated with goat anti-rabbit IgG microbeads for 30 minutes at 4°C, and selected for Nrp-1^high^CD4^+^CD25^+^Tregs and Nrp-1^low^CD4^+^CD25^+^Tregs by MiniMACS separator according to manufacturer's instructions. Isolated cells were cultured in RPMI 1640 supplemented with 10% FCS.

RETRACTED

### 2.4. Sepsis Model

After being anesthetized, a 0.5 cm incision was made on the abdomen of mouse, and the cecum was exposed. The cecum at the designated position between its distal pole and ileocecal junction was ligated for the desirable degree of sepsis: 1/3 for low-grade sepsis, 2/3 for midgrade sepsis, and ligated ileocecal junction for high-grade sepsis. Single puncture was made through the cecum. The diameter of puncture needle was 0.6 mm, and it was used to induce CLP in the experiment. The abdominal incision was closed with simple running sutures. The mice were given a subcutaneous injection of 0.9% sterile saline solution with an amount of 40 mL/kg body weight after CLP.

### 2.5. Experimental Design

150 mice were used to investigate the severity-dependent response between the expressions of Nrp-1 and Foxp-3 of Tregs, and they were divided into five groups: control group, sham group, and three different CLP groups (low-grade, midgrade, and high-grade), with 30 mice in each group. With the optimal degree of sepsis, another 150 mice were employed to observe the time-dependent response between the expressions of Nrp-1 and Foxp-3 of Tregs, and they were divided into five groups: control group and CLP with four interval groups (12, 24, 48, and 72 hours), with 30 mice in each group. The survival time and rate of various groups were recorded.

The optimal grade and time point were used to investigate the impact of Nrp-1 on the negative immunoregulation of Tregs in sepsis. CD4^+^CD25^+^Tregs were further segregated into Nrp-1^high^CD4^+^CD25^+^Tregs and Nrp-1^low^CD4^+^CD25^+^Tregs by MiniMACS separator. They were divided into four groups with the same cell number: control group and CLP with three different subtype Tregs (CD4^+^CD25^+^Tregs, Nrp-1^high^CD4^+^CD25^+^Tregs, and Nrp-1^low^CD4^+^CD25^+^Tregs). They were cocultured with conventional CD4^+^CD25^−^ T cells for 24 hours in a ratio of 1 : 1 and treated with anti-CD3 (5 *μ*g/mL) and anti-CD28 (2 *μ*g/mL) antibody for polyclonal activation of T cells, respectively [14–16]. The proliferative activity, apoptotic rate, and secretive ability (including interferon- (IFN-) *γ* and IL-4) of CD4^+^CD25^−^ T cells and the expression of Foxp-3/CTLA-4/TGF-*β* ^m+^/Nrp-1, apoptotic rate, and secretive ability (including IL-10 and TGF-*β*) of every subtype of Tregs were determined.

RETRACTED

*In vitro*, Nrp-1^high^CD4^+^CD25^+^Tregs were isolated from normal mice spleen and cultured with different doses (including 1, 10, 100, 1000, and 10000 *μ*g/mL) of recombinant Nrp-1 polyclonal antibody in the stimulated LPS (1000 ng/mL) for 24 hours. The demethylation level of Foxp-3-TSDR was determined by demethylation-sensitive RT-PCR, which had been recounted by Tatura et al. [13].

### 2.6. CCK-8 Measurement

The proliferative activity of CD4^+^CD25^−^ T cells was determined by CCK-8 according to protocols provided by the manufacturer. The absorbance was read in microplate reader (Spectra MR, Dynex, Richfield, MN) at OD 450 nm.

### 2.7. Flow Cytometric Analysis

CD4^+^CD25^+^Tregs were stained with FITC-conjugated anti-mouse-CTLA-4, APC-conjugated anti-mouse/rat-TGF-*β* ^m+^, or APC-conjugated anti-mouse/rat-Nrp-1 for 30 minutes at 4°C in the dark based on the same cell number. For determination of intranuclear Foxp-3, CD4^+^CD25^+^Tregs were suspended in 1 mL fixation/permeabilization solution for 2 hours at 4°C in the dark. After washing cells with permeabilization buffer twice, CD4^+^CD25^+^Tregs were stained with FITC-conjugated anti-mouse/rat-Foxp-3 for 30 minutes at 4°C in the dark. After washing CD4^+^CD25^+^Tregs with phosphate-buffered saline (PBS) twice, cells were analyzed with flow cytometer (BD Biosciences, Mountain View, CA). 5 × 10^5^–1 × 10^6^ CD4^+^CD25^+^Tregs or CD4^+^CD25^−^ T cells were washed with PBS twice; cells were suspended in 200 *μ*L binding buffer, followed by 10 *μ*L FITC-conjugated annexin-V to stain for 30 minutes at 4°C or 15 minutes at 25°C in the dark. 300 *μ*L binding buffer and 5 *μ*L PI were added to stain for 5 minutes at 25°C in the dark again, and they were subjected to flow cytometric analysis by flow cytometer.

### 2.8. ELISA Measurement

The supernatants were collected for measuring the levels of IFN-*γ*, IL-4, TGF-*β*, and IL-10 by ELISA kits, strictly according to the manufacturer's protocols. Plates were read in microplate reader at OD 450. The standard concentration curves for IFN-*γ*, IL-4, TGF-*β*, and IL-10 were plotted from 0 to 1000 pg/mL. Examination of all samples was run in quintuplicate.

### 2.9. Statistical Analysis

Data was represented as mean ± standard deviation (SD) and analyzed by SPSS 17.0 software with a one-way ANOVA. Unpaired Student's* t*-test was used to evaluate significant differences between groups. A *P* value of 0.05 or 0.01 was considered statistically significant. Survival rate in septic mice was evaluated by Kaplan-Meier via the log-rank test.

RETRACTED

## 3. Results

### 3.1. Sepsis Markedly Enhanced the Expression of Nrp-1 on CD4^+^CD25^+^Tregs in a Grade- and Time-Dependent Pattern

As shown in Figures 1(a) and 1(e), CD4^+^CD25^+^Tregs were isolated from spleens at 24 hours after CLP, and it was found that, compared with the control group, expressions of Nrp-1 and Foxp-3 of CD4^+^CD25^+^Tregs were significantly promoted by sepsis (*P* < 0.01). Compared with low-grade septic group, the expressions of Nrp-1 and Foxp-3 were further promoted in mid- and high-grade septic groups (*P* < 0.01), and the difference between mid- and high-grade septic groups was not statistically significant (*P* > 0.05). As shown in Figure 1(b), the survival rate of low-, mid-, and high-grade septic groups was 86.67%, 66.67%, and 33.33%, respectively. The differences between them were statistically significant according to Kaplan-Meier analysis (*P* < 0.01). In Figures 1(a), 1(b), and 1(e), we noticed that sepsis promoted the expression of Nrp-1 along with the severity of sepsis and the upregulation of cytoactivity of CD4^+^CD25^+^Tregs. We used midgrade septic model to further observe the time-dependent impact of sepsis on the expression of Nrp-1 and Foxp-3. As shown in Figures 1(c) and 1(f), compared with the control group, the expressions of Nrp-1 and Foxp-3 were significantly promoted at every point after CLP (*P* < 0.01). Compared with 12-hour group, expressions of Nrp-1 and Foxp-3 were markedly enhanced at 24 and 48 hours (*P* < 0.01), but they were downregulated at 72 hours, and the difference between them was not statistically significant (*P* > 0.05). The survival rate of 12-, 24-, and 48-hour groups was 93.33%, 66.67%, and 26.67% (Figure 1(d)), respectively, and the differences between them were statistically significant according to Kaplan-Meier analysis (*P* < 0.01), but the difference between 48- and 72-hour (20%) groups was not statistically significant (*P* > 0.05).

### 3.2. Sepsis Upregulated the Expression of Foxp-3/CTLA-4/TGF-*β* ^m+^ on Nrp-1^high^CD4^+^CD25^+^Tregs

As shown in Figures 2(a), 2(b), and 2(c), midgrade septic model was used to evaluate the impact of Nrp-1 on the negative immunoregulation of Tregs at 24 hours after CLP. Compared with the control group, sepsis significantly upregulated the expression of Foxp-3/CTLA-4/TGF-*β* ^m+^ on CD4^+^CD25^+^Tregs and Nrp-1^high^CD4^+^CD25^+^Tregs (*P* < 0.01), but the expression of Foxp-3/CTLA-4/TGF-*β* ^m+^ on Nrp-1^low^CD4^+^CD25^+^Tregs was significantly downregulated (*P* < 0.01). Compared with CD4^+^CD25^+^Tregs, expressions of Foxp-3/CTLA-4/TGF-*β* ^m+^ on Nrp-1^high^CD4^+^CD25^+^Tregs were further obviously upregulated (*P* < 0.01).

RETRACTED

### 3.3. Nrp-1^high^CD4^+^CD25^+^Tregs Had the Strongest Resilience to Apoptosis in Sepsis

As shown in Figure 3, with the midgrade septic model at 24 hours, compared with the control group, the apoptotic rates of CD4^+^CD25^+^Tregs and Nrp-1^high^CD4^+^CD25^+^Tregs were markedly reduced (*P* < 0.01), but the apoptotic rate of Nrp-1^low^CD4^+^CD25^+^Tregs was increased (*P* < 0.05). In contrast to CD4^+^CD25^+^Tregs, the apoptotic rate of Nrp-1^high^CD4^+^CD25^+^Tregs was further obviously reduced (*P* < 0.01).

### 3.4. Nrp-1^high^CD4^+^CD25^+^Tregs Showed the Strongest Ability to Secrete Inhibitory Cytokines

As shown in Figure 4, with the midgrade septic model at 24 hours, CD4^+^CD25^+^Tregs, Nrp-1^high^CD4^+^CD25^+^Tregs, and Nrp-1^low^CD4^+^CD25^+^Tregs were cocultured with CD4^+^CD25^−^ T cells for 24 hours in a ratio of 1 : 1, respectively. The production of IL-10 and TGF-*β* was significantly increased from CD4^+^CD25^+^Tregs and Nrp-1^high^CD4^+^CD25^+^Tregs compared with that of the control group (*P* < 0.01), especially for Nrp-1^high^CD4^+^CD25^+^Tregs as compared with that of CD4^+^CD25^+^Tregs (*P* < 0.01). However, IL-10 and TGF-*β* levels were significantly descended in Nrp-1^low^CD4^+^CD25^+^Tregs (*P* < 0.01).

### 3.5. Nrp-1^high^CD4^+^CD25^+^Tregs Had the Strong Ability to Inhibit the Proliferation and Increase the Apoptosis of CD4^+^CD25^−^ T Cells

CD4^+^CD25^+^Tregs, Nrp-1^high^CD4^+^CD25^+^Tregs, and Nrp-1^low^CD4^+^CD25^+^Tregs were isolated from the midgrade septic model at 24 hours and cocultured with conventional CD4^+^CD25^−^ T cells for 24 hours with a ratio of 1 : 1, respectively. Compared with the control group, the proliferation (Figure 5(a)) of CD4^+^CD25^−^ T cells was significantly suppressed, and the apoptosis (Figures 5(b) and 5(c)) of CD4^+^CD25^−^ T cells was significantly increased when cocultured with CD4^+^CD25^+^Tregs and Nrp-1^high^CD4^+^CD25^+^Tregs (*P* < 0.01), but the proliferation of CD4^+^CD25^−^ T cells was obviously upregulated, and the apoptosis of CD4^+^CD25^−^ T cells was obviously downregulated, when cocultured with Nrp-1^low^CD4^+^CD25^+^Tregs (*P* < 0.01). Compared with CD4^+^CD25^+^Tregs, the proliferation of CD4^+^CD25^−^ T cells was further significantly inhibited, and the apoptosis of CD4^+^CD25^−^ T cells was further significantly increased when cocultured with Nrp-1^high^CD4^+^CD25^+^Tregs (*P* < 0.05 or 0.01).

### 3.6. Nrp-1^high^CD4^+^CD25^+^Tregs Inhibited Secreting Cytokines of CD4^+^CD25^−^ T Cells

As shown in Figure 6, CD4^+^CD25^+^Tregs, Nrp-1^high^CD4^+^CD25^+^Tregs, and Nrp-1^low^CD4^+^CD25^+^Tregs were, respectively, isolated from the midgrade septic model at 24 hours and cocultured with CD4^+^CD25^−^ T cells for 24 hours in a ratio of 1 : 1. In comparison to the control group, secretion of IFN-*γ* of CD4^+^CD25^−^ T cells was decreased, but release of IL-4 was increased when cocultured with CD4^+^CD25^+^Tregs (*P* < 0.05). Nrp-1^high^CD4^+^CD25^+^Tregs significantly suppressed the secretion of IFN-*γ* and IL-4 from CD4^+^CD25^−^ T cells as compared with the control group and CD4^+^CD25^+^Tregs (*P* < 0.05 or 0.01). The formation of IFN-*γ* and IL-4 from CD4^+^CD25^−^ T cells was significantly upregulated when cocultured with Nrp-1^low^CD4^+^CD25^+^Tregs (*P* < 0.01).

RETRACTED

### 3.7. Recombinant Nrp-1 Polyclonal Antibody Downregulated the Demethylation Level of Foxp-3-TSDR

As shown in Figure 7,* in vitro*, the demethylation level of Foxp-3-TSDR in Nrp-1^high^CD4^+^CD25^+^Tregs was significantly increased in the stimulated LPS compared with control group for 24 hours (*P* < 0.01); recombinant Nrp-1 polyclonal antibody had an obvious ability to downregulate the demethylation level of Foxp-3-TSDR, and in a dose-dependent manner, especially 10000 *μ*g/mL (*P* < 0.05 or 0.01).

## 4. Discussion

Foxp-3, which is still the main intracellular marker for identification of Tregs, is a distinctive transcriptional factor of Tregs, and it is also critical for their function, differentiation, and maintenance [11, 13, 26]. Our previous study demonstrated that a significantly increased expression of Foxp-3 in Tregs was positively correlated with the mortality of burn-induced septic mice [14–17]. Recently, Nrp-1, which was highly expressed on natural Tregs but lowly expressed on induced Tregs and not expressed on CD4^+^CD25^−^ cells, is a good marker to distinguish natural and induced Tregs [20–24]. More interestingly, another study showed a population of Nrp-1^+^Tregs in human lymph nodes together with the positive expression of Foxp-3 that inhibited the proliferative activity of T cells [27]. In the current study, we first reported that sepsis* per se* markedly promoted the expression of Nrp-1 on CD4^+^CD25^+^Tregs in a grade- and time-dependent manner, the expression of Nrp-1 on Tregs was obviously correlated with the expression of Foxp-3 and the mortality of CLP-induced septic mice, and Nrp-1 had prevented ability to preserve the negative immunoregulation of Tregs in sepsis.

It has been known that immune dysfunction of CD4^+^ T-lymphocytes was one of the primary cellular mechanisms in sepsis-induced immunosuppressive state [28]. Immediate observation of specimens from spleen, thymus, and lung in septic patients who died in intensive care units, or those from murine CLP model, showed a profound, progressive, apoptosis-induced loss of adaptive immunocytes, thereby resulting in a decrease in ability of producing antibodies and clearing life-threatening pathogens [6, 7, 29–31]. It is well known that the activated CD4^+^ T cells can mainly differentiate into Th1 and Th2, and they mainly produced IFN-*γ* and IL-4, respectively [29]. A shift to Th2 response was noted to be corroborated sepsis-induced immunosuppression, and the secretion of Th1 associated cytokines was thereby impaired, and, on the other hand, the secretion of Th2 associated cytokines was increased during sepsis, and these phenomena were obviously correlated with the outcome of septic complications [7, 31]. T cells are anergic when they respond to their specific antigens, which are identified as failure to proliferate or secrete cytokines [30]. In the present study, the results suggested that Nrp-1^high^CD4^+^CD25^+^Tregs had the strongest ability to inhibit the proliferation and increase the apoptosis, as well as inhibiting the cytokine secretion of CD4^+^CD25^−^ T cells, but Nrp-1^low^CD4^+^CD25^+^Tregs had opposed ability on CD4^+^CD25^−^ T cells; thus, we conjectured that Nrp-1^low^CD4^+^CD25^+^Tregs had a potential ability to prevent cellular immunosuppression in sepsis.

RETRACTED

In the development of sepsis, Tregs can mainly inhibit the activation of T-lymphocytes, especially CD4^+^ T-lymphocytes through various suppressive mechanisms, including inhibitory cytokines (such as IL-10 and TGF-*β*) and cell-to-cell contact (such as CTLA-4 and TGF-*β* ^m+^), inhibition of cytolysis (especially granzymes), downregulation of metabolic disruption, and suppression of maturation and function of antigen presenting cells, as well as upregulation of antiapoptotic ability [12, 14–17]. Accumulated evidence has shown that a combination of Foxp-3, CTLA-4, TGF-*β* ^m+^, and inhibitory cytokines (IL-10 and TGF-*β*) might serve as active markers for Tregs in the process of sepsis [6, 7, 13, 29, 30]. We used a midgrade septic model reproduced 24 hours after CLP to investigate the impact of Nrp-1 on the negative immunoregulation of Tregs in the setting of sepsis. It was found that sepsis could obviously upregulate the negative immunoregulation of CD4^+^CD25^+^Tregs and Nrp-1^high^CD4^+^CD25^+^Tregs, especially Nrp-1^high^CD4^+^CD25^+^Tregs, but downregulated the negative immunoregulation of Nrp-1^low^CD4^+^CD25^+^Tregs, which correlated with the expressions of Foxp-3/CTLA-4/TGF-*β* ^m+^ and the apoptotic ability, as well as the secretion of IL-10 and TGF-*β*.

RETRACTED

We have reported that the percentage and stability of Tregs were higher in septic patients and mice septic models than in those without sepsis. A reduction in the percentage and stability of Tregs was accompanied by an improvement in survival rate and immune dysfunction of T-lymphocytes in septic mice [14–17]. It has been documented that the stability of Tregs includes the stability of Foxp-3 expression and negative immunoregulatory function in sepsis, which is crucially dependent on the demethylation status of the Foxp-3-TSDR [13]. In the current study, we found that recombinant Nrp-1 polyclonal antibody could downregulate the demethylation of Foxp-3-TSDR in the presence of LPS; thus, Nrp-1 could represent a new potential therapeutic target, at least via regulating the stability of Tregs, for the study of immune regulation in sepsis.

## 5. Conclusion

In conclusion, the expression of Nrp-1 on CD4^+^CD25^+^Tregs was upregulated in sepsis. Foxp-3/CTLA-4/TGF-*β* ^m+^ of Nrp-1^high^CD4^+^CD25^+^Tregs were significantly upregulated by septic challenge. Nrp-1^high^CD4^+^CD25^+^Tregs showed strong resilience to apoptosis and cytokine secretive ability in sepsis, and they possessed a strong ability to inhibit the proliferation and increase the apoptosis, as well as secreting cytokines of CD4^+^CD25^−^ T cells. Recombinant Nrp-1 polyclonal antibody had the ability to downregulate the demethylation of Foxp-3-TSDR in the presence of lipopolysaccharide (LPS). Nrp-1^high^CD4^+^CD25^+^Tregs might exhibit primary negative immunoregulation in sepsis, and Nrp-1 could represent a new potential therapeutic target for the study of immune regulation in sepsis.

## Figures and Tables

**Figure 1:** The grade- and time-dependent responses between sepsis and the expression of Nrp-1 in splenic CD4^+^CD25^+^Tregs. The results showed the effects of various severities of sepsis on the expression of Nrp-1 in splenic CD4^+^CD25^+^Tregs at 24 hours after CLP ((a), (e)). The grade-dependent impact between sepsis and the 24-hour survival rate (b). The effects of midgrade sepsis on the expression of Nrp-1 of splenic CD4^+^CD25^+^Tregs at 12, 24, 48, and 72 hours after CLP ((c), (f)). The time-dependent response between sepsis and the 72-hour survival rate (d). Data was represented as mean ± standard deviation (SD) and analyzed by SPSS 17.0 software with a one-way ANOVA, *n* = 4 per group (*P* < 0.01). The survival rate was analyzed by Kaplan-Meier via the log-rank test, *n* = 30 per group (*P* < 0.05 or *P* < 0.01).

**Figure 2:** Sepsis markedly upregulated the expression of Foxp-3/CTLA-4/TGF-*β* ^m+^ on Nrp-1^high^CD4^+^CD25^+^Tregs. Midgrade septic model at 24 hours after CLP was used to investigate the effect of Nrp-1 on the negative immunoregulation of Tregs in sepsis. The expressions of Nrp-1 and Foxp-3 ((a), (c)) and CTLA-4 and TGF-*β* ^m+^ ((b), (c)) were subjected to flow cytometric analysis by flow cytometer. Data was represented as mean ± standard deviation (SD) and analyzed by SPSS 17.0 software with a one-way ANOVA, *n* = 4 per group (*P* < 0.01).

RETRACTED

**Figure 3:** Nrp-1^high^CD4^+^CD25^+^Tregs showed the strongest resilience to apoptosis in sepsis. The apoptotic rate of Tregs was analyzed with annexin-V-FITC/PI flow cytometry at 24 hours after midgrade sepsis. Data was represented as mean ± standard deviation (SD) and analyzed by SPSS 17.0 software with a one-way ANOVA, *n* = 4 per group (*P* < 0.05 or *P* < 0.01).

**Figure 4:** Nrp-1^high^CD4^+^CD25^+^Tregs showed the strong ability to secrete cytokines. Sepsis could markedly enhance the release of IL-10 and TGF-*β*. Data was represented as mean ± standard deviation (SD) and analyzed by SPSS 17.0 software with a one-way ANOVA, *n* = 4 per group (*P* < 0.01).

**Figure 5:** Nrp-1^high^CD4^+^CD25^+^Tregs showed the strong ability to inhibit the proliferation and increase the apoptosis of CD4^+^CD25^−^ T cells. Three different subtype Tregs groups (CD4^+^CD25^+^Tregs, Nrp-1^high^CD4^+^CD25^+^Tregs, and Nrp-1^low^CD4^+^CD25^+^Tregs) were cocultured with CD4^+^CD25^−^ T cells for 24 hours in a ratio of 1 : 1; the proliferative ability of CD4^+^CD25^−^ T cells (a) and apoptotic rate of CD4^+^CD25^−^ T cells ((b), (c)) were determined. Data was represented as mean ± standard deviation (SD) and analyzed by SPSS 17.0 software with a one-way ANOVA, *n* = 4 per group (*P* < 0.05 or *P* < 0.01).

**Figure 6:** Nrp-1^high^CD4^+^CD25^+^Tregs showed the strong ability to suppress cytokine release of CD4^+^CD25^−^ T cells. Three different subtype Tregs (CD4^+^CD25^+^Tregs, Nrp-1^high^CD4^+^CD25^+^Tregs, and Nrp-1^low^CD4^+^CD25^+^Tregs) were cocultured with CD4^+^CD25^−^ T cells for 24 hours, and the secretion of IFN-*γ* and IL-4 of CD4^+^CD25^−^ T cells was measured. Data was represented as mean ± standard deviation (SD) and analyzed by SPSS 17.0 software with a one-way ANOVA, *n* = 4 per group (*P* < 0.05 or *P* < 0.01).

**Figure 7:** Recombinant Nrp-1 polyclonal antibody markedly downregulated the demethylation of Foxp-3-TSDR in the stimulated LPS at 24 hours in a dose-dependent manner. Data was represented as mean ± standard deviation (SD) and analyzed by SPSS 17.0 software with a one-way ANOVA, *n* = 4 per group (*P* < 0.05 or *P* < 0.01).
